# Key Technologies of Lightweight Materials for New Energy Vehicles Based on Ant Colony Algorithm

This article has been retracted.

**DOI:** 10.1155/2022/1617814

**Published:** 2022-06-17

**Authors:** Lin Mei, Li Xiaoke

**Affiliations:** College of Physics and Engineering Technology, Chengdu Normal University, Chengdu, Sichuan 611130, China

## Abstract

From the perspective of the new energy vehicle, application of lightweight technology can effectively improve the endurance level of new energy vehicles and promote the steady improvement and rapid development of China's new energy vehicle industry. By keeping in view the importance of lightweight effect of new energy vehicles, in this paper, we have carried out an in-depth analysis of key contents such as new materials, battery weight, carbon fiber technology, and structural design technology in the process of lightweight development of new energy vehicles. Furthermore, this paper introduces the pseudorandom proportional rule to improve the selection method of the seed solution, makes appropriate random disturbance to the center of the pheromone distribution, and reforms the standard deviation of the pheromone distribution. Taking the lightweight of new energy vehicle doors as an example, this paper verifies the new energy vehicle lightweight algorithm based on ant colony algorithm. It is found that the improved continuous domain basic ant colony algorithm is superior to the other two algorithms and it has the capacity to solve optimization problems and has the advantages of high reliability.

## 1. Introduction

Climate change, environmental degradation, energy consumption, and other issues are important concerns that threaten the world's ability to develop sustainably today, and they have long been the focus of the international community's attention and efforts. WAS has undertaken research on regional and national Life Cycle (LCA) policies in Europe, North America, China, Japan, and other areas and nations [1–4]. The European Parliament endorsed the final emission reduction report published earlier this year, which was adopted in April 2019. North America has made significant contributions to environmental background activities, as well as possible data and methodologies. In collaboration with China Tsinghua University, China Automobile Center, and the Society of Automotive Engineers, several new standards, such as the LCA carbon emission group standard and the 2019 China Low Carbon Action Plan Research Report, were released. To realize the technical aim of zero carbon emissions through the development of hydrogen energy, improvements in transportation efficiency, and intelligent design, old Toyota, Mazda, and the Ministry of Economy, Trade, and Industry, among others, have revised their LCA policy viewpoints. In this context, the vehicle sector, which is the second greatest emitter of carbon dioxide in the world, has a substantial impact on the long-term development of the environment and its sustainability. Since 2016, China has also surpassed the United States as the world's largest vehicle consumer market and manufacturer. It has the responsibility and the obligation to investigate the impact of the development of the automobile industry on the sustainable development of the environment, and through appropriate development strategies and measures, the automobile industry not only brings convenience to people's travel but also ensures that the environment is not burdened with an increased burden of pollution [5–9].

Usually, new energy vehicles are powered by batteries, hybrid power, ethanol, hydrogen energy, and other forms of renewable energy as these vehicles have a number of inherent benefits over traditional fuel vehicles. During the driving phase of the vehicle, these vehicles either do not emit CO or emit less CO and particulate matter compared to what the vehicle would otherwise emit. Following implementation, new energy will emerge in a more environmentally friendly manner during the stages of production, mining, and recycling, and the number of emissions throughout the whole life cycle will continue to be decreased. New energy vehicles have been intensively created as a result of this policy and technology, and a great deal of research has been done on the corresponding lightweight body structure, body material, battery frame, battery energy density, and safety. The selection and implementation of technology have demonstrated a development pattern that differs from that of traditional fuel-powered transportation [10–12].

Automotive lightweight technology is a multi-industry technology type that involves joint breakthroughs in many disciplines, including the automobile manufacturing industry, the material technology industry, the design and development industry, and the process optimization industry. Moreover, it has the potential to drive a rapid improvement in the production level of relevant parts and components in China's vehicle manufacturing business, as well as a gradual improvement in the ability of autos to innovate. Current government policy identifies automobile lightweight development technology (ALDT) as one of the development technology routes in key areas, and it proposes that the value of more instructive, more guiding, and strategic planning significance be determined in accordance with the development status of China's automobile industry (ACI). As a result, the discussion and research on the core technologies of lightweight new energy vehicles presented in this paper have both theoretical and practical significance [13–19].

It is a type of swarm intelligence algorithm, and it was originally designed to tackle the optimization issue of discrete variables. In recent years, there has been an increase in interest in continuous domain ant colony algorithms, as well as improvements in research and application [20–25]. According to some researchers, the ACOR algorithm is a framework for solving the optimization issue in the continuous domain. It is distinguished by the use of a Gaussian distribution to simulate the pheromone distribution in the algorithm. Other researchers have proposed that the mutation technique in ABC be used to update the global pheromone in the ACOR algorithm. It was decided to create a new ABC-ACOR algorithm. At the moment, the example verification of the continuous domain ant colony method is primarily concerned with the pure mathematical optimization problem, with the constraints being taken into consideration only in passing [26–30].

This paper addresses the shortcomings of the basic ant colony algorithm in the continuous domain such as poor local exploration ability, poor stability, and insufficient constraint processing and then applies the improved continuous domain ant colony algorithm to the lightweight problem of new energy vehicles to demonstrate the effectiveness of the enhancements made. The algorithm's dependability plays a part in boosting the lightweight study of new energy vehicles, which is important in a number of ways.

The rest of the paper is arranged as given below.

Key technologies for lightweight new energy vehicles are described in detail in Section 2 of the paper. Additionally, a detailed description about development of the material for the problem in hand is provided. The proposed model that is primarily based on the ant colony optimization algorithm is reported along with its numerous section and supportive mathematical equations. Simulation results are presented in Section 4 where it is evident that the proposed scheme is an ideal solution. Lastly, summary of the overall work presented in this paper is presented.

## 2. Key Technologies for Lightweight New Energy Vehicles

As we all know, batteries, motors, and electronic control systems are the primary components of new energy vehicles. Even while this method may significantly improve the application capability as well as the technical level of new energy vehicles, it also significantly increases the number of new energy vehicles on the road. In new energy cars, the weight of the vehicle has a significant impact on the vehicle's performance in terms of power, braking, safety, endurance, and battery use. According to data analysis, reducing the weight of new energy cars by 20 percent can successfully enhance battery life by 5 to 10% while also saving between 15 and 120 percent on battery expenses. It can also help to lower the amount of new energy cars that are used on a daily basis. In order to lower the weight of modern energy vehicles, it is critical that they be built more efficiently. Starting with the vehicle itself, lightweight technology for new energy vehicles works toward the aim of reduced nominal density, which is achieved by decreasing the weight of the vehicle. The quality of the new energy vehicle in the same volume state improves as the nominal density of the new energy vehicle increases. However, it is difficult to change the battery energy density of the vehicle in a short period of time, and the battery life of the new energy vehicle cannot be guaranteed. Applications are in the areas of safety, performance, and electrical energy. Conclusion: by reducing the nominal density of new energy vehicles, the light weight of new energy vehicles has the potential to considerably improve their overall endurance.

### 2.1. Development of New Materials and Putting Them into Mass Use

The entire vehicle equipment for new energy vehicles is made up of a variety of components. Following the molding process, the weight of any part is a fixed parameter. The overall weight parameter of the car can be calculated by summing up the weight parameters of all of the car's components. Many sections and components of modern energy vehicles are currently comprised of steel materials, resulting in a significant increase in the overall weight of the vehicle. As a result, using new materials to replace traditional steel materials in the manufacture of automobile parts and the provision of related devices are very effective in reducing the overall weight of new energy cars. The ultimate purpose of ongoing development and research into new materials, high-performance automotive plastics, carbon fiber composite materials, aluminum alloy structures, magnesium alloy structures, and other materials is to meet the mechanical properties, physical parameters, and structural design requirements of new energy vehicles in their normal use. On a bigger scale, the new energy vehicle market can benefit from better development and application of demand and safety requirements. For example, in 2016, Chery New Energy Vehicle independently developed an aluminum alloy skeleton structure and applied this structure to the mass market production of pure electric vehicles, reducing the total weight of this type of vehicle by approximately 30% compared to other vehicles of the same type, and it was finally warmly welcomed by the market as a result of its superior performance characteristics.

### 2.2. Optimization of Battery Weight

The single capacity of the battery for the new energy vehicle is predetermined. For the new energy vehicle to operate normally and smoothly, it is frequently essential to integrate thousands of battery cells with fixed capacities to make a comprehensive battery pack structure, which can take several months to complete. The overall mass of the vehicle is frequently greater than a few hundred kilograms, and this element of the weight accounts for a significant amount of the total weight of the vehicle. The optimization of the new energy vehicle's battery weight is therefore a key step in the process of reducing the overall weight of the new energy vehicle. In this process, the actual capacity of a single battery can be broken through by increasing the capacity of a single battery of the new energy vehicle, allowing the total number of battery cells required by the new energy vehicle to be reduced on the assumption that the predetermined capacity of the battery has been reached. The number of times it is used consequently lowers the overall quality of the battery pack as a whole. When attempting to reduce the weight of the battery, it is possible to improve the capacity of the battery cell through innovative design and transformation, as well as optimization of the battery capacity parameters, and to optimize the cell structure size of the new energy battery cell, so that the cell size does not affect the capacity of the battery. The discharge power of the battery is guaranteed to increase as the discharge power of the battery rises in voltage. The battery life of a new energy vehicle can be significantly increased by improving the internal structure of the battery cell, without having to change the total number of batteries used in the vehicle. Examples include Nissan automobiles, which frequently reduce the total weight of new energy vehicles by optimizing the internal structural size of their battery cells, which may often be reduced by approximately 80 kg.

### 2.3. Using Carbon Fiber Technology

Using artificial synthesis technology, carbon fiber technology arranges organic fibers such as flake or broken graphite crystals in a specific organizational structure in the axial direction in order to achieve strong mechanical properties and, ultimately, to meet the mechanical structure requirements of the material. According to relevant studies, carbon fiber material parts are approximately one-fourth the weight of steel material parts for parts of the same size and structure, but the tensile performance of carbon fiber materials is approximately seven times that of steel materials, and the mechanical performance test indicators are far superior to those of steel materials. It outperforms the parameters required by modern energy vehicles in terms of structural and mechanical qualities, for example, while at the same time, the corrosion resistance of carbon fiber materials and the shielding function of the battery construction considerably outperform those of comparable steel materials of the same size. The use of carbon fiber technology in new energy cars can therefore ensure that the car's original performance indicators stay maintained while also achieving the lightweighting target that was set for it. As far as new energy vehicle producers throughout the world are concerned, the usage of carbon fiber technology is still in the early stages of research and investigation at this point. BMW, for example, has grown to a high level of proficiency in the utilization of carbon fiber technology. Carbon fiber materials have been used extensively in the development of the BMW i3 series. When compared to steel materials, carbon fiber materials have contributed approximately 300 kg to the weight reduction of the car. Other automobile manufacturers have failed to achieve the goal of mass production through the application of carbon fiber technology; however, the successful application of BMW's carbon fiber technology in mass production can provide solid support for the use of carbon fiber technology in new energy vehicles in order to reduce the overall weight of the vehicle. It can also help to advance the development of carbon fiber technologies in the future. At the moment, the carbon fiber technology developed in China has achieved relatively positive results in the application of new energy vehicles. As a result of their technological research and development as well as their market practice, several vehicle manufacturing firms have implemented carbon fiber materials into the mass production of automobiles, resulting in a reduction in the actual total weight of the automobile. The reduction of around 50% will aid in the improvement of the battery life of future energy vehicles. According to relevant statistics, the real battery life of new energy cars can be increased to as much as 440 kilometers by incorporating carbon fiber technology into the design.

### 2.4. Optimal Structural Design Technology

Optimizing the structural design of the complete vehicle is a critical step in the process of developing new energy vehicles that are lightweight. This can be accomplished by optimizing the structural architecture of the vehicle with the goal of reducing the overall weight of the vehicle. Under normal circumstances, improvements and optimizations to the vehicle structure can be achieved primarily through three approaches. First, without changing the strength parameters of the vehicle itself, the number of new energy vehicle parts used to achieve the goal of reducing the weight of the vehicle can be reduced through the simplified design of the entire vehicle structure; second, without changing the new energy vehicle parts used to achieve the goal of reducing the weight of the vehicle, the vehicle's overall weight can be reduced. Lastly, in the process of new energy vehicle production and layout, the compact structural design of the parts is utilized to minimize the number of vehicles produced under the premise of overall performance. This is accomplished by shrinking the size of the auto parts in order to achieve a lighter vehicle. The overall volume is reduced in order to meet the goal of being lightweight.

### 2.5. Material Selection Requirements for New Energy Vehicles

In the future, the combination of numerous materials is more likely to be used in automotive lightweight material solutions in order to take full advantage of various materials. Additional current research hotspots and trends in lightweight materials include lowering the cost of materials through technological advancement, reducing the use of scarce metals, increasing the utilization rate of materials and developing new materials that are more environmentally friendly and recyclable. In order to achieve the primary goal of material selection for new energy vehicles based on the fundamental characteristics of materials, the manufacturing process requirements, and the overall performance requirements of new energy vehicles, it is necessary to use suitable materials for suitable parts on the vehicle's body. Several steel kinds are available, each with a different strength range, making them appropriate for use in the design of all covering and structural components. Materials of low density, such as aluminum, magnesium, plastic, and carbon fiber, are appropriate for use in lightweight construction. The specific stiffness index (the ratio of elastic modulus to density) can be used for a variety of applications. When a part is simply subjected to homogeneous uniaxial stress, steel outperforms aluminum and magnesium, while carbon fiber outperforms all of the other materials in terms of strength.

According to existing research and development expertise, steel has excellent crash resistance as well as processing technology and cost benefits. As a result, steel has been widely utilized in automobile body parts as well as suspension and steering system components for many years now. While aluminum alloy material has a lower elastic modulus than regular steel, it has a higher extrusion resistance than conventional steel. It has the potential to increase the rigidity of complicated cross-sectional components while also providing considerable advantages in collision energy absorption, which can result in lower material consumption and component costs. The level is excellence. When utilized in automobile bumpers, engine cooling fans, interiors, and other areas where organic polymer compounds are used to reduce the weight of the vehicle and absorb collision energy, plastics are considered to be among the most effective materials available. Materials with greater energy-absorbing qualities, such as foamed aluminum and woven composite materials, are being employed in the construction of automobile structures.

At the moment, the majority of automotive manufacturers look to BMW as a model for the development of lightweight automobiles, and BMW firms have further strengthened their position as leaders in the development and transformation of automobile lightweight technology. In conjunction with the progressive rise in vehicle placement, the transition from high-strength steel materials to aluminum alloy materials, and ultimately the application of carbon fiber and other polymer composite materials, has occurred. In conjunction with the further maturation of BMW's new 7 Series and BMW Group's new energy vehicle research and development technologies, the proportion of BMW series cars utilizing composite materials has reached an all-time high. The BMW 3 Series is a popular model in the market because it is an important representative of the automotive manufacturer and because it is a typical model that is well accepted. The carbon fiber and polymer composite material technology has been profoundly influenced by the mass production of composite materials, which has had a significant impact on the lightweighting process. When it comes to the upper half of the body, composite materials are most effective when applied efficiently. When the lower frame structure of aluminum alloy is combined with the battery structure, it assures strong collaboration between the new higher material and the frame design after the lower design has been refined, resulting in a weight reduction of 300 kg for the entire vehicle.

## 3. Proposed Model

We first introduce the CDACO algorithm based on ACOR. The continuous domain optimization problem can be written in the following general form:

(1) $$\begin{array}{c} \underset{x\in D}{\min}f\left(x\right)\in R, \end{array}$$

where *x* is an *n*-dimensional real vector, *f*(*x*) is the objective function, and *D* is the *n*-dimensional search space.

Suppose there are *m* groups of ant colonies, each group contains *n* ants, one group of ant colonies can just correspond to a point in the *n*-dimensional search space *D*, and one ant is only responsible for the search of one dimension. The position of a group of ant colonies in *D* can represent a group of solutions, and a total of *m* groups of solutions are obtained, that is, *x*_1_=(*x*_*i*1_, *x*_*i*2_, ⋯, *x*_in_); these *m* groups of solutions are based on the target. The function values are arranged in ascending order, and the evaluation value *Q*_*i*_ of the solution is given by

(2) $$\begin{array}{c} Q_{i}=\frac{1}{lm\sqrt{2\pi }}e^{{\left(i-1\right)}^{2}/2l^{2}-m^{2}}. \end{array}$$

The probability *p*_*i*_ of each solution to be selected is obtained:

(3) $$\begin{array}{c} p_{i}=\frac{Q_{i}}{\sum_{j=1}^{m}Q_{j}}. \end{array}$$

And the probability density function of the solution component *x*_*ij*_ is

(4) $$\begin{array}{c} \alpha_{ij}\left(x\right)=\frac{1}{\sqrt{2\pi }\sigma_{ij}}c^{{\left(x-\mu_{ij}\right)}^{2}/2\sigma_{ij}^{2}}, \end{array}$$

(5) $$\begin{array}{c} \sigma_{ij}=\mu \sum_{s=1}^{m}\frac{\left|x_{ij}-x_{sj}\right|}{m-1}. \end{array}$$

We sample around each solution component *x*_*i*_ of the seed solution *x*_*ij*_ according to the Gaussian distribution described by (4) and (5) and generate a new solution component *x*_*ij*_′

(6) $$\begin{array}{c} x_{ij}^{\prime }=\mu_{ij}+\text{Random}\cdot \sigma_{ij}, \end{array}$$

where Random denotes the random number.

Then we have

(7) $$\begin{array}{c} \Omega =\left\{\begin{array}{c} g_{i}\left(x\right)\leq 0,1,2,\cdots ,l,\\ h_{i}\left(x\right)\leq 0,j=t+1,t+2,\cdots ,rm\\ l_{k}\leq x_{k}\leq u_{k},\;k=1,2,\cdots ,n. \end{array}\right., \end{array}$$

The CDACO algorithm makes reasonable use of the fundamental concept of ant colony foraging, and it fully exploits the positive and negative feedback mechanisms of pheromones to its maximum potential. The algorithm is simple to implement and offers a high level of efficiency. The CDACO method, on the other hand, is prone to falling into a local optimum, having low algorithm stability, and only partially digesting constraints.

In the ACS method, the pseudorandom proportional rule is introduced to select the seed solution, and the specific operation is carried out in accordance with

(8) $$\begin{array}{c} x_{i}=\left\{\begin{array}{c} \arg\max\left(Q_{i}\right),q\leq q_{0},\\ K,q>q_{0}, \end{array}\right. \end{array}$$

where *x_i_* is input, he Gaussian distribution is used as the solution component *μ*_*ij*_, and the distribution model of the pheromone is represented by the center of the Gaussian distribution of the pheromone; as a result, during the operation of sampling to generate a new solution, the new solution components are frequently concentrated. It is quite simple to achieve a local optimum in the vicinity *μ*_*ij*_. Because of this, while selecting some new solutions, the distribution center *x*_*ij*_=*μ*_*ij*_ is affected in the right manner, as indicated in the following equation:

(9) $$\begin{array}{c} \mu_{ij}=x_{ij}+F\left(x_{uj}-x_{vj}\right), \end{array}$$

where *x*_*uj*_, *x*_*vj*_ are the *j*th solution components in the other two solutions randomly selected. *F* ∈ [0.4, 0.9] is a random parameter that can control the size of the disturbance.

In order to deal with the limitations, the CDACO algorithm employs the penalty function technique, which will have a detrimental impact on the optimization process. When dealing with restrictions, it is vital to keep certain infeasible options on mind because the best solution is more likely to be found towards the boundary of the problem. The DCPM technique is created in order to deal with the constraints imposed by the CDACO algorithm, and the variable *W*(*x*) is used to measure the extent to which the solution *x* breaks the restrictions:

(10) $$\begin{array}{c} W\left(x\right)=\sum_{j=1}^{r}c_{j}\left(x\right). \end{array}$$

For *g*_*i*_(*x*) ≤ 0, we let *c*_*j*_(*x*)=max{0, *g*_*j*_(*x*)}; then, we have

(11) $$\begin{array}{c} c_{j}\left(x\right)=\left\{\begin{array}{cc} \left|h_{j}\left(x\right)\right|, & \left|h_{j}\left(x\right)\right|>h_{j\min},\\ 0, & \text{else.} \end{array}\right. \end{array}$$

If *W*(*x*)=0, then *x* fully complies with the constraints; the larger *W*(*x*), the greater the degree of violation of the constraints by *x*. Use *p*_max_ to represent the maximum proportion of infeasible solutions that are allowed to exist.

We name the improved algorithm IACO, and the IACO algorithm flow is as follows:

1. Randomly generate *m* sets of solutions in *D,* and initialize the algorithm parameters; the initial number of iterations *w*=0, and the upper limit of the number of iterations is *M.*
2. *w*=*w*+1.
3. Prepare each group of solutions by calculating the objective function value of each group, sorting them, and then calculating the evaluation value and selection probability of each group of answers.
4. According to the method given by (8), combined with (2) and (3), select the seed solution *x*_*i*_.
5. According to *x*_*i*_, *k* groups of new solutions are generated.
6. Process the constraints and get the updated *m* solutions.
7. If *w* > *M*, stop the iteration and output the optimal solution; otherwise, go to step (2) to continue the iteration.

## 4. Results

In order to verify the application effect of the IACO algorithm in practical engineering problems, the proposed algorithm is used to carry out a lightweight design of the body structure of a new energy battery vehicle. The finite element model of the whole energy vehicle is shown in Figures 1 and 2.

When optimizing side impact and roof collapse, the surrogate model is employed in this paper, which is discussed in detail later. The lightweight design process for a car body based on the IACO algorithm is comprised mostly of the four steps listed:

1. Create a simulation finite element model, specify optimization targets, constraints, and design variables, and then run the simulation.
2. The average grid element size of the vehicle finite element model is 10 mm, and the total number of elements in the model is 1047681. The curb weight of the vehicle is 2 213.9 kg, and the average grid element size of the vehicle finite element model is 10 mm.
3. The laws GB20071-2006 “Occupant Protection in Vehicle Side Accident” mandated the development of a finite element model of a vehicle side collision, which is seen in Figure 3. It is estimated that the simulation time is 150 ms, and the performance indicators investigated are as follows: the maximum deformation speed of the lower ribs of the dummy, the maximum deformation speed of the B-pillar, the maximum deformation speed of the door, the force on the abdomen of the dummy, and the force on the pelvis of the dummy. The simulation time is 150 ms, and the performance indicators investigated are as follows: the plate thicknesses of the 15 components that were shown to be the most susceptible to side impact were chosen as design variables.
4. The roof crush simulation model is developed in accordance with the requirements of the American standard FMVSS216. The force of the pressure plate when the crushing depth of the pressure plate is 127 mm has been selected as the performance index to be used. Upon completion of the safety evaluation, the maximum force of the top pressure rebound is determined to be greater than 50 kN. A total of ten plate thicknesses associated with top crushing were selected as design factors.
5. Carry out the experimental design in the problem design space, obtain the output response by finite element simulation, and construct the appropriate surrogate model for each collision scenario, in addition to assessing the accuracy of the surrogate models. In this work, the Kriging surrogate model technology is used, and the accuracy of the model is updated using the target-oriented sequence sampling technology, which is described in detail below.
6. First, for each design variable, an experimental design is carried out in order to determine its effects. It is necessary to perform sampling in the design domain using the best Latin hypercube approach available. Check whether the certainty coefficient of each surrogate model matches the design requirements in order to verify the correctness of each surrogate model. Make it accurate enough to suit the criteria of any further surrogate model applications you may have. The deterministic coefficients of the new surrogate models are all more than 0.9, which satisfies the accuracy requirements and allows the problem to be addressed by further optimization after the revision.
7. To tackle the constrained optimization problem, the IACO algorithm is utilized as a solution method.
8. In addition, the validity of the optimization solutions is checked by the use of finite element simulations.

In order to simulate the structural performance, substitute the optimized solution after rounding into the finite element simulation model. As long as the constraint performance index of each working condition is satisfied, the total mass of the 25 kinds of plates participating in the optimization under the two working conditions is reduced from 48.35 to 42.31, a reduction of 6.04 kg, and the lightweight effect reaches 15.92 percent, according to the results. The usefulness of the algorithm suggested in this research in reducing the weight of the body of a new energy vehicle is demonstrated in this study.

Further, this paper compares the performance of different algorithms for lightweight effect on ten models, as shown in Figure 4, and it can be seen that the IACO algorithm is significantly better than other algorithms.

The maximum deformation speed of the B-pillar is also investigated in this paper using different methods on 10 models, as depicted in Figure 5 of the article. This clearly demonstrates how much better the IACO algorithm is compared to the other algorithms.

## 5. Conclusion

In this paper, we have conducted an in-depth examination of key contents such as new materials, battery weight, carbon fiber technology, and structural design technology which are used in the lightweight development of new energy cars. Future development paths for automobile lightweight technology and new energy vehicle lightweighting in the international community are being charted out for the time being. Additionally, we have introduced a pseudorandom proportional rule to improve the method of selecting the seed solution, introduced appropriate random disturbance to the center of the pheromone distribution, and modified the standard deviation of the pheromone distribution, all of which contribute to improved performance. This research examines the lightweight of new energy vehicle doors as an example and the lightweight algorithm for new energy vehicles based on the ant colony algorithm is proven. In this study, it is discovered that the modified continuous domain basic ant colony method outperforms the other two algorithms and its application to optimization problems has the advantage of high reliability.

In future, application of the proposed model can be extended to other areas of the automobiles as well.

## Figures and Tables

**Figure 1:** The finite element model of the whole vehicle.

**Figure 2:** The finite element model of the whole vehicle.

**Figure 3:** Finite element model of vehicle side collision.

**Figure 4:** Comparison of lightweight effects of different algorithms.

**Figure 5:** Comparison of B-pillar effects of different algorithms.

## Data Availability

The data used to support the findings of this study are available from the corresponding author upon request.
